RETRACTED

# Methyltransferase like 7B is upregulated in sepsis and modulates lipopolysaccharide-induced inflammatory response and macrophage polarization

**DOI:** 10.1080/21655979.2022.2068892

**Published:** 2022-05-21

**Authors:** Dan Huang, Hai Yan

**Affiliations:** a Clinical Medical College of Chengdu Medical College, Chengdu, China; b Department of Critical Care Medicine, The First Affiliated Hospital of Chengdu Medical College, Chengdu, China; c Department of Gastrointestinal Surgery, The First Affiliated Hospital of Chengdu Medical College, Chengdu, China

**Keywords:** METTL7B, sepsis, macrophages, inflammation, polarization

## Abstract

Macrophages play a critical role in the regulation of the inflammatory responses in sepsis. Methyltransferase like 7B (METTL7B) has been implicated in several pathophysiological conditions. Nevertheless, the potential engagement of METTL7B in sepsis remains to be elucidated. In this study, we retrieved transcriptomic profile data of septic patients and healthy donors and compared the expression level of METTL7B between septic patients and healthy controls. We also collected septic patient samples to analyze METTL7B expression via RT-qPCR. Murine bone marrow-derived macrophages (BMDMs) were isolated and treated with incremental doses of LPS as an *in vitro* cell model. METTL7B was overexpressed or knocked down in BMDMs, and lipopolysaccharide (LPS)-mediated inflammatory cytokines production and macrophage polarization were evaluated. We found that METTL7B was upregulated in the blood and peripheral blood mononuclear cells (PBMC) of septic patients, which also showed a significant diagnostic potential for sepsis. In BMDMs, METTL7B was induced in a time and dose-dependent manner by LPS. Modulating the expression level of METTL7B could regulate LPS-mediated inflammatory cytokines production and macrophage polarization. The functional role of METTL7B was also validated in a septic mouse model. Our findings indicate that METTL7B is implicated in the immunopathogenesis of sepsis through modulating macrophage-mediated inflammatory responses. METTL7B may serve as a potential diagnostic and therapeutic target for sepsis.

## Highlights

- METTL7B is upregulated in the peripheral blood and PBMCs of sepsis patients
- METTL7B promotes inflammatory responses and M1 macrophage polarization
- Silencing METTL7B attenuated M1 macrophage polarization *in vitro and in vivo*

## Introduction

As a major public health burden, sepsis is characterized by multiple organ dysfunction induced by polymicrobial infection [1]. The uncontrolled infection triggers host immune responses, which subsequently initiates an escalating cascade of inflammatory reactions and organ damages [2]. Despite the application of antimicrobial agents and medical interventions, sepsis remains as one of the leading causes of death worldwide in intensive care units [3]. Early diagnosis is crucial in the management of sepsis since prompt treatment can prevent the aggravation of the pathophysiological progression of severe sepsis. Therefore, identification of promising diagnostic and therapeutic biomarkers is of great value for the management of sepsis.

RETRACTED

Macrophages participate in both innate and adaptive immunity, and they are recognized as a major player in modulating the inflammatory responses during sepsis [4,5]. Mounting evidence has demonstrated that macrophages seem to play different roles in different stages of sepsis [4]. Macrophages can be polarized toward proinflammatory (M1) and anti-inflammatory (M2) phenotypes depending on the combination and strength of stimulation signals [6]. In the early stage of sepsis, M1 macrophages accumulate significantly, leading to the massive production of proinflammatory factors such as interleukin 1β (IL-1β), IL-6, tumor necrosis factor-α (TNF-α) and inducible nitric oxide synthase (iNOS). However, at the later stage of sepsis, macrophages primarily exhibit an M2 phenotype and act as anti-inflammatory regulators [4,7]. Accordingly, modulating the plasticity and polarization phenotype of macrophages has a direct impact on the outcome of sepsis. It is of great clinical significance to figure out the molecular mechanism underlying macrophage polarization in sepsis.

Methytransferase like proteins (METTL) are a diverse family of proteins characterized by the presence of methyltransferase like domains and a structurally-conserved binding domain for S-adenosyl methionine [8,9]. METTL7B, a member of mammalian METTL family, is localized on chromosome 12. Accumulating evidence has demonstrated that METTL7B is implicated in several pathophysiological conditions, such as cancers [10–13], nonalcoholic steatohepatitis lipid metabolism [14], severe preeclampsia [15] and microbial infection [16]. However, the biological functions of METTL7B remain to be explored, and whether METTL7B is implicated in the progression of sepsis is largely unknown.

In this study, we first analyzed transcriptomic datasets (GSE95233 and GSE133822) containing septic patients and healthy donors. We found that METTL7B was significantly upregulated in septic patients, and therefore hypothesized that the upregulation of METTL7B contributes to the progression of sepsis. Using blood samples and peripheral blood mononuclear cells (PBMC) of sepsis patients, we validated the upregulation of METTL7B in sepsis. Since macrophages are implicated in the inflammatory progression of sepsis, we then explored the potential role of METTL7B in macrophage polarization by gain-of-function and loss-of-function experiments. Based on the cell model of LPS-stimulated murine bone marrow-derived macrophages (BMDMs) and the animal model of sepsis, our study unveiled a novel role of METTL7B in the polarization of macrophages, which may contribute to the inflammatory progression of sepsis.

RETRACTED

## Materials & methods

### Gene expression profiles

Two gene expression datasets (GSE95233 and GSE133822) were retrieved from GEO database (http://www.ncbi.nlm.nih.gov/geo). A total number of 51 septic shock patients and 22 healthy donors were included in GSE95233 dataset [17]. The blood samples from septic shock patients were collected twice at two different time points. However, considering the samples’ uniformity, we only analyzed the data from the blood samples collected on Day1. The GSE133822 dataset contains 33 human sepsis and 22 normal PBMC samples [18]. Differential gene expression analysis was performed using the edgeR package in R software. Significantly differentially expressed genes (DEGs) were identified using the following criteria: adjusted P value < 0.05 and the |log2FC (fold change) | > 1. The expression value of *METTL7B* was obtained from the series_matrix.txt of GSE95233 and GSE133822, and then presented in dot plot.

### Patient samples

A total of 30 patients who met Sepsis-3 criteria [1] and 30 healthy individuals as controls were recruited with the approval of the Ethics Committee of the First Affiliated Hospital of Chengdu Medical College, and informed consent was obtained from all patients. Exclusion criteria: patients who were pregnant; patients who had organ (including heart, liver and kidney) dysfunctions; patients who were diagnosed with malignant tumors; patients who were infected with human immunodeficiency virus; and patients who had autoimmune diseases. The clinical characteristics of enrolled patients were summarized in Table 1. Peripheral blood samples were collected from those subjects using EDTA tubes at the time of intensive care unit admission. The blood samples were divided into two parts: one was directly used as whole blood, and the other one was used to isolate PBMC. PBMCs were isolated from the peripheral blood samples by density gradient centrifugation as previously described [19]. Briefly, 10 ml of blood samples were diluted 1:1 with phosphate-buffered saline, and then were carefully underlaid with Ficoll-Paque (ThermoFisher, USA) at room temperature. Subsequently, the samples were centrifuged at 800 g for 30 minutes and the PBMC layer was harvested with a sterile pipette.

RETRACTED

**Table 1.** Clinical characteristics of sepsis patients and healthy controls

Characteristics	Sepsis patients (n = 30)	Healthy controls (n = 30)
Gender, Male	17	20
Age, years	46(33–62)	43(31–58)
APACHE II score	16.2(13.7–22.3)	NA
SOFA score	9.1(6.3–15.2)	NA
WBC, x10^9^/L	13.2(10.3–23.5)	7.1(4.8–9.6)
CRP, mg/L	124.0(65.3–199.8)	NA
Infection site, no. of patients		
Respiratory tract	13	NA
Gastrointestinal tract	11	NA
Urinary tract	4	NA
Other	3	NA
Bacteremia	24	NA
Length of ICU stay, days	8 [3–15]	NA
Death, no. of patients	3	NA

Data are expressed as median (interquartile range); APACHE II score: acute physiology, age and chronic health evaluation II score; SOFA score: sequential organ failure assessment score; WBC: white blood cells; CRP: C-reaction protein; NA: not applicable.

### Bone marrow-derived macrophages (BMDM)

Wild-type male C57BL/6 J mice (6–8 weeks) were maintained at the Clinical Medical College of Chengdu Medical College. Murine BMDM were isolated from C57BL/6 J mice in accordance with the protocols as described previously [20]. In brief, bone marrow cells were flushed out from the tibias and femurs of mice using PBS supplemented with 3% fetal bovine serum (FBS; Gibco, USA), and then filtered through a 70 µm cell strainer. Subsequently, cells were cultured in Dulbecco’s modified Eagle medium containing 10% FBS, 100 U/mL penicillin, 100 μg/mL streptomycin (Gibco, USA) and 10 ng/ml M-CSF (Sigma-Aldrich, USA) for 7 days. The adherent cells were finally washed with cold PBS and then harvested and cultured in DMEM for the following experiments. For measuring *METTL7B* expression, BMDMs were plated in 12-well plates or 6-well plates for 24 h, and then stimulated with 10 ng/ml or 100 ng/ml lipopolysaccharide (LPS, Sigma-Aldrich). Cells were collected at the indicated time points and used in the analysis of *METTL7B* mRNA and protein expression. The animal studies were approved by the Animal Management and Use Committee of the Clinical Medical College of Chengdu Medical College.

### Cell transfection

The siRNA targeting *METTL7B* (si-*METTL7B*) was purchased from Ribobio (Guangzhou, China). The lentivirus (with green fluorescent protein tag) encoding the *METTL7B* (Lv-*METTL7B*) sequences was provided by GeneChem (Shanghai, China). The isolated BMDMs were seeded in 6-well plates. After growing for 24 h, cells were transfected with 100 nM si-*METTL7B* or si-control using Lipofectamine 3000 (Invitrogen, USA). Similarly, 200 µL Lv-*METTL7B* or Lv-control (multiplicity of infection = 30) and HitransG infection enhancer reagent (GeneChem) were added into each well to overexpress *METTL7B* in BMDMs. Lentivirus transduction efficiency was evaluated under fluorescence microscope 48 h after infection.

RETRACTED

### Quantitative real-time polymerase chain reaction (qRT-PCR)

Total RNA of the blood samples and cells were extracted using Trizol reagent (Invitrogen, USA), followed by reverse transcription into cDNA with HiScript® II Q RT SuperMix (Vazyme, China). Next, qRT-PCR was performed with AceQ® Universal SYBR qPCR Master Mix (Vazyme) in a LightCycler® 480 PCR System (Roche). The relative RNA levels were normalized against GAPDH and 2^–ΔΔCt^ method was used for analysis. The primer sequences used in this experiment were listed in Table 2.

**Table 2.** The primer sequences for qRT-PCR

Gene	Forward	Reverse
m_GAPDH	TCTGACGTGCCGCCTGGAGA	CAGCCCCGGCATCGAAGGTG
m_METTL7B	CCTGCCTAGACCCAAATCCC	AAACCGCTCATATTGGAGGTG
m_IL-1β	CCTCGTGCTGTCGGACCCATA	CAGGCTTGTGCTCTGCTTGTGA
m_IL-6	TAGTCCTTCCTACCCCAATTTCC	TTGGTCCTTAGCCACTCCTTC
m_TNF-α	CCTGTAGCCCACGTCGTAG	GGGAGTAGACAAGGTACAACCC
m_iNOS	CAGCTGGGCTGTACAAACCTT	CATTGGAAGTGAAGCGTTTCG
m_Arg1	CTCCAAGCCAAAGTCCTTAGAG	GGAGCTGTCATTAGGGACATCA
h_GAPDH	CTGGGCTACACTGAGCACC	AAGTGGTCGTTGAGGGCAATG
h_METTL7B	GCAACCGCAAGATGGAGAG	GATTTGGGTCTAGGCAGGTGA

m_murine; h_human.

### Western blotting

Total proteins were extracted from BMDMs by lysing the cells in cold RIPA buffer (Beyotime Biotechnology, China) supplemented with protease and phosphatase inhibitor Cocktail (MedChemExpress, China) for 15 mins. After centrifugation, the supernatant containing total protein lysate was quantified by a BCA Protein assay kit (Beyotime Biotechnology, Shanghai, China). 20 µg of protein samples were separated by 10% sodium dodecyl sulfate polyacrylamide gel (SDS-PAGE) and then transferred onto polyvinylidene difluoride membranes. Subsequently, after blocking with 5% nonfat milk for 1 h at room temperature, the membranes were then incubated with primary anti-*METTL7B* (ab243710, Abcam, UK) and GAPDH antibody (Proteintech, China) overnight at 4°C. The membrane was washed 3 times with TBST and further incubated with HRP-linked secondary antibody (Cell Signaling Technologies, MA, USA) at room temperature for 1 hour. Then the membrane was washed 4 times with TBST, and the protein bands were developed using an enhanced chemiluminescence kit (Santa Cruz, TX, USA). The protein bands were photographed on a gel imager system (Bio-Rad, Hercules, CA, United States). The densitometry analysis was performed with Image J software (Bethesda, MD, USA).

### Enzyme linked immune-sorbent assay (ELISA)

For the measurement of cytokines production, pre-transfected BMDMs were seeded in 12-well plates and cultured overnight. Then the cells were challenged with 100 ng/ml LPS for 6 h. The levels of IL-1β, IL-6 and TNF-α in the culture supernatants were detected using ELISA kits (R&D Systems, USA) according to the manufacturer’s instructions.

RETRACTED

### Flow cytometry analysis

Macrophage polarization was assessed by flow cytometry based on CD38 and CD206 staining. BMDMs were first blocked by Anti-Human IgG Fc antibody (1:200, Abcam, USA) for 15 mins, and then stained with antibodies against CD38 (1:200, Abcam, USA) and CD206 (, 1:300, Abcam) to differentiate M1 and M2 phenotypes, respectively. The relative surface staining of CD38 and CD206 was analyzed on BD FACS CantoTM II Flow Cytometer (BD Biosciences, USA).

### Animal model of sepsis induction

8-week-old male mice were injected intraperitoneally with 30 mg/kg LPS. The mock group was injected with equal volume of PBS. The rescue group was injected with LPS and 0.1 mg/kg si-METTL7B or si-NC. Each group contains 5 mice. After 48 h, BMDMs samples were collected from the tibias and femurs, and the inflammatory cytokine expression was analyzed by qRT-PCR and the polarized phenotype of macrophage was analyzed by flow cytometry.

### Statistical analysis

All data were analyzed by SPSS 18.0 statistical software and expressed as mean ± standard deviation (SD). Data analysis by student’s t-test was used to evaluate the differences between two groups. One-way analysis of variance (ANOVA) was used for evaluating the differences among multiple groups, and Tukey’s post hoc test for performed for pairwise comparison. * *P* < 0.05, ** *P* < 0.01, ***P < 0.001 indicated a significant difference.

## Results

In this study, we found that METTL7B was upregulated in the blood and PBMC samples of sepsis patients in published transcriptomic dataset, which was validated in the clinical samples of septic patients. Based on LPS-induced BMDMs *in vitro* model, we showed that METTL7B silencing attenuated the inflammatory polarization of M1 macrophages, while METTL7B overexpression promoted M1 polarization. The effect of METTL7B silencing was further evaluated in a septic mouse model. Our finding suggests that the upregulation of METTL7B may contribute to the progression of sepsis.

### The upregulation of METTL7B in the peripheral blood and PBMCs of sepsis patients

To examine the relative expression of METTL7B in sepsis patients, we first extracted and analyzed the transcriptomic data from GSE95233 and GSE133822 datasets [17,18]. There are 51 blood samples from sepsis patients and 22 blood samples from healthy controls in GSE95233, while GSE133822 contains 33 sepsis and 22 normal PBMC samples. As a result, the mRNA level of METTL7B was significantly elevated in the blood samples (Figure 1a) and in the PBMCs of septic patients (Figure 1b). We also collected blood samples and isolated PBMCs from 30 septic patients and 30 healthy controls to validate the findings by qRT-PCR. As expected, the results were consistent with the observation in GSE dataset (Figure 1 c and d). To evaluate the diagnostic potential of METTL7B expression in sepsis, we performed the receiver operating characteristics (ROC) analysis in the cohort. As shown in Figure 1e, for blood METTL7B levels, the cutoff value at 1.885 had a sensitivity 86.7% with the area under the curve (AUC) of 0.841. For METTL7B levels in PBMCs, the cutoff value at 1.37 had a sensitivity 90% with the AUC of 0.878 (figure 1f). These results suggest that increased METTL7B levels in the blood and PBMCs have a great diagnostic value for sepsis.

RETRACTED

**Figure 1.** The expression and diagnostic value of *METTL7B* in patients with sepsis. (a) The relative expression of METTL7B in the blood of sepsis patients and healthy controls based on the dataset GSE95233; (b) The relative expression of METTL7B in PBMCs of sepsis patients and healthy controls based on the dataset GSE133822; (c) The relative expression of METTL7B in the blood samples of 30 sepsis patients and 30 healthy control by qRT-PCR; (d) The relative expression of METTL7B in the PBMCs isolated from 30 sepsis patients and 30 healthy control by qRT-PCR; (e) The diagnostic value of blood METTL7B level analyzed by ROC curve; (f) The diagnostic value of METTL7B levels in the PBMCs analyzed by ROC curve. *** P < 0.001, analyzed by student’s t test.

### LPS induces METTL7B expression in murine BMDMs

Considering LPS is a frequently used inducer in murine septic models both *in vivo* and *in vitro*, we next investigated whether LPS affected METTL7B expression in murine BMDMs. Murine BMDMs were stimulated by LPS (10 ng/ml and 100 ng/ml) for 12 h. As shown in Figure 2 a and b, both the mRNA and protein levels of METTL7B were remarkably increased in a dose-dependent manner. In addition, we also treated BMDMs with LPS for different durations, and found that METTL7B mRNA and protein levels were gradually elevated with an increased treatment time, which peaked at 24 h (Figure 2 c and d). However, at 48 h METTL7B expression level showed a marginal drop. Thus, these findings revealed that LPS treatment induce the expression of METTL7B mRNA and protein in murine BMDMs in a dose and time-dependent manner.

**Figure 2.** METTL7B expression is induced by LPS in a time and dose-dependent manner in BMDMs. (a-b) BMDMs were treated with 10 ng/ml or 100 ng/ml LPS for 12 h. The expression of METTL7B was determined by qRT-PCR and Western blotting; Data are the summary of 3 independent experiments; (c-d) BMDMs were treated with 100 ng/ml LPS for 0, 3, 6 h,12, 24 and 48 h. The expression of *METTL7B* was determined by qRT-PCR and Western blotting. Data are the summary of 3 independent experiments. ANOVA was used for evaluating the differences among multiple groups. *, **and*** indicate P < 0.05, 0.01 and 0.001, respectively. All experiments were repeated 3 times.

RETRACTED

### Silencing of METTL7B attenuates the production of proinflammatory cytokines in LPS-stimulated BMDMs

To further explore the functional role of METTL7B in LPS-stimulated inflammatory cytokines production in murine BMDMs, we silenced METTL7B in murine BMDMs using siRNA targeting METTL7B. The transfection of si-METTL7B showed efficient knockdown effect on both METTL7B mRNA and protein (Figure 3 a and b). We then challenged BMDMs with LPS, which significantly upregulated IL-1β, IL-6 and TNF-α mRNA levels. However, METTL7B knockdown significantly attenuated the upregulation of these genes (Figure 3c). Moreover, we also performed ELISA to determine the protein levels of these inflammatory cytokines in the culture supernatants, and similar results were observed as shown in Figure 3d-f. Thus, METTL7B upregulation is indispensable for the proinflammatory cytokine production in BMDMs upon LPS stimulation.

**Figure 3.** METTL7B silencing attenuated LPS-induced pro-inflammatory cytokines in BMDMs. (a-b) Validation of METTL7B knockdown efficiency of si-METTL7B by qRT-PCR and Western blotting, Data are the summary of 3 independent experiments; (c) BMDMs were treated with 100 ng/ml LPS for 6 h. The mRNA levels of IL-6, TNF-α and IL-1β were determined by qRT-PCR, all experiments were repeated 3 times and n = 5 technical replicates in group; (d-f) After stimulation with 100 ng/ml LPS for 6 h, IL-6, TNF-α and IL-1β levels in the culture supernatants of BMDMs were determined by ELISA, all experiments were repeated 3 times and n = 5 technical replicates group. Student’s t test was used for two-group comparison, and ANOVA was used for evaluating the differences among multiple groups. * and ** indicate P < 0.05 and 0.01, respectively.

### METTL7B overexpression augments pro-inflammatory cytokine production in BMDMs

A lentivirus encoding METTL7B sequences was used for METTL7B overexpression in murine BMDMs. After the viral transduction, METTL7B expression was significantly increased at both mRNA and protein levels (Figure 4 a and b). In contrast to the results of METTL7B knockdown, the overexpression of METTL7B augmented pro-inflammatory cytokine production in BMDMs upon LPS challenge (Figure 4c-f). Therefore, a high level of METTL7B promotes pro-inflammatory cytokine production.

**Figure 4.** Overexpression of METTL7B augments LPS-induced pro-inflammatory cytokine production in BMDMs. (a-b) Validation of METTL7B overexpression after lentiviral transduction by qRT-PCR and Western blotting. Data are the summary of 3 independent experiments; (c) BMDMs were treated with 100 ng/ml LPS for 6 h. The mRNA levels of IL-6, TNF-α and IL-1β were determined by qRT-PCR, all experiments were repeated 3 times and n = 5 technical replicates per group; (d-f) After stimulation with 100 ng/ml LPS for 6 h, IL-6, TNF-α and IL-1β levels in the culture supernatants of BMDMs were determined by ELISA, all experiments were repeated 3 times and n = 5 technical replicates per group. Student’s t test was used for two-group comparison, and ANOVA was used for evaluating the differences more than three groups. * and ** indicate P < 0.05 and 0.01, respectively.

RETRACTED

### *The functional role of METTL7B in LPS-mediated macrophage polarization* in vitro

Given that METTL7B regulates LPS-induced proinflammatory cytokines in BMDMs, we subsequently examined whether METTL7B regulates macrophage polarization. As expected, LPS treatment greatly increased the expression of iNOS (M1 phenotype marker), while Arg1 (M2 phenotype marker) expression was significantly down-regulated in murine BMDMs (Figure 5 a and b), which is consistent with the previous report [21]. However, compared to the control group, METTL7B silencing dramatically reduced iNOS expression and elevated Arg1 expression, whereas METTL7B overexpression showed the opposite effects (Figure 5 a and b).

**Figure 5.** The relative expression level of METTL7B regulates LPS-mediated macrophage polarization. BMDMs were transfected with si-METTL7B or transduced with Lv-METTL7B, and then challenged with 100 ng/ml LPS for 6 h. Cells were then stained with antibodies targeting M1 macrophage marker CD38 or M2 macrophage marker CD206. (a-b) The mRNA levels of iNOS and Arg-1 were determined by qRT-PCR. Data are the summary of 3 independent experiments; (c) METTL7B silencing decreases the proportion of M1 macrophages upon LPS induction as determined by CD38 staining; (d) METTL7B silencing increases the proportion of M2 macrophages upon LPS induction as determined by CD206 staining; (e) Overexpression of METTL7B increases the proportion of M1 macrophages upon LPS induction as determined by CD38 staining; (f) Overexpression of METTL7B decreases the proportion of M2 macrophages upon LPS induction as determined by CD206 staining. Data are the summary of 3 independent experiments. ANOVA was used for evaluating the differences among multiple groups. * and ** indicate P < 0.05 and 0.01, respectively. All experiments were repeated 3 times and n = 5 per group.

To further analyze the polarized phenotype, we then examined the protein level of cell surface marker of different macrophage phenotypes (CD38 for M1 and CD206 for M2) using flow cytometry in si-METTL7B or Lv-METTL7B treated BMDMs upon LPS stimulation. METTL7B silencing caused a significant reduction of CD38+ BMDMs (Figure 5c) and increase of CD206+ BMDMs (Figure 5d), whereas METTL7B overexpression resulted in an increase of CD38+ BMDMs (Figure 5e) and decrease of the proportion of CD206+ BMDMs (figure 5f) upon LPS stimulation. It is noteworthy that in the absence of LPS challenge, METTL7B expression level did not affect BMDM polarization. Taken together, our data indicate that a high expression level of METTL7B could drive LPS-mediated macrophage polarization toward proinflammatory M1 phenotype *in vitro*, while METTL7B silencing could promote M2 polarization.

RETRACTED

### Silencing of METTL7B impaired M1 macrophage polarization in LPS induced sepsis mouse model

To further validate the role of METTL7B in macrophage polarization *in vivo*, mice were injected intraperitoneally with LPS or with equal volume of PBS, together with si-METTL7B or si-NC (n = 5 in each group). After 48 h, we collected the BMDMs, and qRT-PCR analysis showed that LPS treatment induced METTL7B upregulation, and si-METTL7B suppressed METTL7B expression in both LPS or PBS treated groups (Figure 6a). LPS treatment significantly upregulated IL-1β, IL-6 and TNF-α mRNA levels and METTL7B knockdown significantly attenuated the upregulation of these genes (Figure 6b). Furthermore, METTL7B silencing caused a significant reduction of the percentage of CD38+ BMDMs (Figure 6c) and an increase of CD206+ BMDMs (Figure 6d) in LPS challenged group, while no effect was observed in the groups without LPS challenge. In summary, these data indicate that METTL7B upregulation contributes to the inflammatory cytokine production and M1 macrophage polarization in LPS-induced sepsis mouse model.

**Figure 6.** Silencing METTL7B attenuated LPS-induced M1 macrophage polarization in septic mouse model. (a) Mice were injected intraperitoneally with LPS or with equal volume of PBS, together with si-METTL7B or si-NC (n = 5 in each group). After 48 h, BMDMs were isolated and qRT-PCR analysis showed that LPS induces METTL7B upregulation, and si-METTL7B suppresses METTL7B expression in both LPS or PBS treated groups. (b) The relative level of IL-1β, IL-6 and TNF-α mRNA levels were determined by qRT-PCR in isolated BMDMs. (c) METTL7B silencing decreases the proportion of M1 macrophages upon LPS induction as determined by CD38 staining; (d) METTL7B silencing increases the proportion of M2 macrophages upon LPS induction as determined by CD206 staining. n = 5 mice in each group. ANOVA was used for evaluating the differences among multiple groups. * and ** indicate P < 0.05 and 0.01, respectively.

RETRACTED

## Discussion

METTL7B is a poorly characterized member of the METTL family, which was originally discovered as a Golgi related methyltransferase [22]. Despite that METTL7B has been implicated in the progression of several human cancers [11–13], little is known about the role of METTL7B in the pathogenesis of sepsis. In this study, we found that METTL7B expression was upregulated in the blood and PBMC samples of sepsis patients through bioinformatics analysis, which was validated in the clinical samples of 30 septic patients and healthy controls. Furthermore, we also demonstrated that METTL7B levels both in the blood and PBMCs had a great diagnostic value for sepsis, indicating that METTL7B may serve as a potential biomarker for sepsis. LPS-induced cell model is a frequently used *in vitro* model to investigate the molecular mechanism of sepsis. Thereby, we challenged BMDMs with LPS to study the functional role of METTL7B in macrophages. Consistent with the findings in the clinical samples, LPS stimulation significantly induced METTL7B expression in a time and dose-dependent manner in murine BMDMs. The above finding collectively suggest that the upregulation of METTL7B may contribute to the progression of sepsis.

In the early stage of sepsis, the excessive activation of innate immune cells, including macrophages, results in a cytokine storm characterized by excessive production of proinflammatory factors [23]. Mounting evidence has highlighted a vital role of macrophage polarization in the immunopathogenesis of sepsis [24,25]. Wang et al. recently found that Growth Differentiation Factor 3 (GDF3) strongly suppresses M1 polarization while facilitating M2 polarization *in vivo* and *in vitro*, thereby protecting against lethal sepsis [19]. Arora et al. reported that the ATP Binding Cassette Subfamily F Member 1 (ABCF1) can reduce the mortality of endotoxemia mice through promoting M2 polarization [26]. Additionally, a previous study also demonstrated that adoptive transfer of *ex vivo* programed M2 macrophages is beneficial to the survival of septic mice [27]. Accumulation of M1 macrophages can contribute to the clearance of pathogens, but prolonged M1 polarization leads to tissue and organ damages [7,28]. Instead, M2 macrophages are essential in tissue repair and resolution of inflammation [7]. Hence, it is of great clinical significance to explore the underlying modulatory mechanisms of macrophage polarization during sepsis. Achieving a balanced polarization between pro-inflammatory M1 and anti-inflammatory M2 macrophages would be beneficial to the remission of sepsis.

RETRACTED

In the present study, we showed that *in vitro* silencing of METTL7B dramatically reduced the secretion of proinflammatory cytokines and promoted the polarization of BMDMs toward M2 phenotype upon LPS stimulation, while METTL7B overexpression led to the opposite consequences. Interestingly, METTL7B silencing failed to influence BMDM phenotype in the absence of LPS stimulation, indicating that METTL7B could only regulate the process of macrophage phenotype only when the macrophage polarization is initiated. Our findings indicate that METTL7B upregulation may contribute to the progression of sepsis via promoting the inflammatory phenotype of macrophage. However, the underlying mechanisms by which METTL7B tailors the inflammatory responses and polarization in macrophages remain to be further investigated.

Undoubtedly, there are some limitations of our present work. As an RNA modification enzyme, METTL7B has been shown to regulate cell cycle in tumor progression [11], epithelial-mesenchymal transition [12], and appears to be engaged in the regulation of inflammatory signaling pathways via Janus Kinase 1 (JAK1) [29,30].Therefore, whether METTL7B modulates inflammatory responses by targeting JAK1 needs to be further studied. Besides, the functional roles of METTL7B in LPS-induced endotoxemia mice and cecal ligation and puncture model remain to be explored. In addition, this study only investigated the role of METTL7B in murine BMDMs. The potential engagement of METTL7B in regulating other immune cells still needs to be clarified. Lastly, the detailed mechanisms how METTL7B modulates macrophage phenotypic remain to be investigated in future studies.

## Conclusion

In summary, our study demonstrated that METTL7B is upregulated in the blood and PBMCs of sepsis patients, which may contribute to the immunopathogenesis of sepsis. Based on LPS-induced murine BMDMs, we further showed that METTL7B expression level modulates LPS-induced inflammatory responses and macrophage polarization *in vitro*. Our study unveiled a novel role of METTL7B in modulating macrophage polarization, which may serve as a potential target for the management of sepsis.

## Data Availability

The data is available from the corresponding author on reasonable request.
